# Analysis of Anesthesia Effect of Dexmedetomidine in Clinical Operation of Replantation of Severed Finger

This article has been retracted.

**DOI:** 10.1155/2021/3822450

**Published:** 2021-12-13

**Authors:** Tongsheng Xu, Xiaodong Chen, Xin Li, Mingzhu Wang, Meng Wang

**Affiliations:** Wuxi 9th People's Hospital, Wuxi, China

## Abstract

Brachial plexus block commonly used in finger replantation has the advantages of simple operation, small side effects, and stable circulation, but it has inherent problems such as imperfect block range, slow onset of anesthesia, and short maintenance time of anesthesia. In order to explore the reliable clinical anesthesia effect, this paper uses experimental investigation methods to study the effect of dexmedetomidine in clinical surgery of replantation of severed fingers. Moreover, this paper uses comparative test methods, uses statistical methods to process test data, and uses intuitive methods to display test results. Finally, this paper verifies the reliability of dexmedetomidine in replantation of severed finger through comparative analysis and verifies that the anesthesia method proposed in this paper has certain user satisfaction through parameter survey.

## 1. Introduction

One of the most frequent surgeries in surgery is the replantation of severed fingers. The sensitive technical operation challenges in the replantation of severed fingers have been successfully handled thanks to the microscopic advancement of surgical technology, considerably improving the replantation of severed fingers survival rate [1]. The complexity, length of time, and high intensity of the severed finger replantation procedure, on the other hand, put the patient's surgical tolerance to the test [2]. As a result, developing a proper anesthetic strategy to increase the anesthetic effect is critical for the operation's successful completion. The brachial plexus block, which is often used in finger replantation, offers the benefits of being easy to administer, having few side effects, and providing consistent circulation. It does, however, have flaws such as a limited block range, a sluggish onset of anesthesia, and a short duration of anesthesia. These will make the patient awake, restless, or experience limb discomfort, among other things, causing significant disruption to the procedure and perhaps jeopardising its flawless conclusion [3]. Sedative analgesics such as remifentanil and dexmedetomidine have been demonstrated in studies to improve the impact of local nerve block and extend the duration of analgesia and have therefore become important adjuvants during surgical anesthesia. The conventional dose of remifentanil combined with dexmedetomidine anesthesia has a good anesthetic effect in clinical applications, but at the same time, drug-related side effects are strong, and even excessive sedation of patients occurs, which is not conducive to patient safety [4]. Therefore, the selection and development of a suitable anesthesia plan are of great significance in the replantation of severed fingers.

General anesthetic, local infiltration anesthesia, and brachial plexus block are the most used anesthetic procedures for finger replantation at the moment. General anesthesia can address the need for a longer operation duration for severed finger replantation while also providing a superior anesthetic effect. There are, however, a variety of general anesthetic medicines that might produce hemodynamic abnormalities. Furthermore, extended general anesthesia may lead to significant consequences such aspiration pneumonia, delayed recovery, postoperative nausea and vomiting, hypoventilation, and acute atelectasis. Furthermore, studies have shown that using general anesthesia for upper limb surgery increases the risk of deep vein thrombosis while simultaneously increasing the expense of general anesthesia. As a result, in the replantation of severed fingers, basic general anesthesia is seldom employed. Local infiltration anesthetic, on the other hand, is not suited for long-term hand surgery since it cannot break during the procedure and alleviate the tourniquet discomfort. The brachial plexus is composed of cervical C5--8 and T1 nerve roots, which mainly innervate the sensation and movement of the upper limbs, shoulders, and chest. In comparison to general anesthesia, brachial plexus block is easier to administer, requires less anesthetic medication, has a minimal effect on the entire body, maintains stable circulation, and provides prolonged postoperative analgesia compared to local infiltration anesthesia, and the analgesic effect and intraoperative treatment are superior. Because the effect is superior, it is often utilized in hand surgical anesthetic. The brachial plexus may be blocked by a number of routes, including the intermuscular groove, supraclavicular, subclavian, and axillary approaches, as well as the recently described subcoracoid approach block. However, brachial plexus block also has some inherent problems, such as prone to incomplete block, insufficient onset of anesthesia, and insufficient maintenance time of anesthesia, and patients who are awake are prone to fear and cannot cooperate with surgery. How to solve these problems, many explorations and studies have been done at home and abroad. The first is about the selection of puncture points for brachial plexus block and how to improve the operation of brachial plexus block; the second is adding adjuvants to local anesthetics. In order to speed up the onset of nerve block, prolong the block time, and improve the anesthesia effect; the third is what kind of drugs are used for sedation during the operation without putting the patient's respiratory and circulatory systems at risk; and the fourth is what kind of drugs are used for sedation during the operation without putting the patient's respiratory and circulatory systems at risk. The technical issues of brachial plexus surgery have also been overcome thanks to the widespread use of ultrasonography technology in clinics. As a new field of ultrasound application, nerve block anesthesia guided by ultrasound is gradually attracting attention. The previous blind piercing technique and the positioning of the neurostimulator are not only difficult, but also often incompletely blocked. At the same time, they may cause damage to the nerves and surrounding tissues such as blood vessel structure and pleura, so they are gradually eliminated. Ultrasound technology has revolutionized the way nerve blocks are performed. It has a high level of precision and consistency when it comes to nerve block. Ultrasound pictures are easy to understand. The anesthesiologist may puncture the target peripheral nerve in real time while using ultrasound guidance to study the nerve and its surrounding tissue anatomy. The injection process and diffusion range of the anesthetic ensure that the local anesthetic is evenly diffused to the peripheral nerves, so that the local anesthetic can fully penetrate the nerves, which significantly increases the success rate and reduces complications. The currently recognized approach with the highest success rate is the intermuscular sulcus brachial plexus block. According to research, ultrasound-guided intermuscular sulcus nerve blocks may improve the nerve block's safety and efficacy while also lowering the dosage of local anesthetic. Brachial plexus obstruction is no longer a technological issue. It is worth thinking about what kind of medicine is used as intraoperative sedation and what kind of medicine is used as an adjuvant for local anesthetics. Dexmedetomidine (DEX) is a novel and highly selective adrenoceptor agonist.

This paper studies the clinical application effect of dexmedetomidine in the replantation of severed finger and provides a theoretical reference for the anesthesia process of subsequent severed finger replantation.

## 2. Related Work

Dexmedetomidine is a selective *α*2-adrenergic receptor agonist approved by the US Food and Drug Administration for continuous intravenous sedation in intensive care settings. In a preliminary investigation (data not given), injecting 0.25 percent bupivacaine into the nerve dexmedetomidine during the injection of the rat sciatic nerve increased the duration of sensory and motor block [5]. Other studies have found that dexmedetomidine is safe and effective in various intraspinal and regional anesthetics in humans, including intrathecal injection and intravenous local anesthesia. Although dexmedetomidine prolongs and/or exacerbates the peripheral nerve sensory block caused by local anesthetics, the mechanism behind this is yet unknown. Dexmedetomidine is an agonist of the *α*2 adrenergic receptor [6]. The literature [7] found in the in vitro study of frog sciatic nerve conduction with high concentration of dexmedetomidine that the reduction of the compound's action potential is concentration-dependent rather than *α*2 mediated. In vivo and in vitro studies have found that the effect of clonidine, another *α*2 adrenergic receptor agonist, on peripheral nerves may be mediated by blocking the cation current activated by hyperpolarization, rather than due to the agonistic effects of *α*2 adrenergic receptors. In vitro investigations of dexmedetomidine's action in paraventricular nucleus neurons revealed that it works in part by suppressing Ih current [8]. The present investigation seeks to test the hypothesis that the period of dexmedetomidine analgesia rises to the local anesthetic is mediated by Ih current rather than blockage of 1 or 2 adrenergic receptor agonists in a rat model of peripheral nerve block [9]. To lengthen the duration of analgesia, dexmedetomidine combined rat sciatic nerve block delay ropivacaine to block hyperpolarization triggered cationic current [10]. The Ih current is necessary for restoring the resting potential of peripheral nerves. Hyperpolarization is caused by action potentials, and neurons are unable to create new action potentials. As a result, nerves become resistant to additional stimulation. The nerve must recover to its resting potential in order to produce another action potential [11]. This happens at the end of the repolarization process. Nerve prolonged hyperpolarization is caused by blocking the Ih current, and it seems to be more apparent in unmyelinated fibres (pain) than in A fibres (exercise). As a result, inhibiting the Ih current may have a greater impact on pain than on exercise response [12]. The addition of substantial dosages of dexmedetomidine to bupivacaine considerably improved the feeling and mobility of rats with sciatic nerve block, according to the literature [13]. The central analgesic impact of dexmedetomidine is only substantial when bupivacaine is added, disputing the central analgesic effect of dexmedetomidine as a cause for prolonging sensory block duration. Dexmedetomidine alone does not cause considerable sensory or motor block, which is similar to what has been reported with clonidine in laboratory and clinical studies [14].

Replantation of severed finger is a refined and long-term operation. A single intermuscular groove or axillary ropivacaine block is sometimes difficult to meet the needs of replantation surgery. It often causes pain, anxiety, and fear of the patient, resulting in failure of replantation. Continuous nerve block is complicated to operate, inconvenient to manage, high cost, high complication rate, and little practical value. Daily clinical practice proves that clonidine is an *α*2 adrenergic receptor agonist, which can prolong peripheral nerve block duration. Dexmedetomidine is a highly selective *α*2 adrenergic receptor agonist. Therefore, dexmedetomidine is an auxiliary drug for nerve block. When it is used in conjunction with local anesthetics, it can enhance the effect of blocking sensory and motor, shortening the time of sensory block and prolonging the time of sensory and motor recovery [15].

General anesthetic, brachial plexus block, and local infiltration anesthesia are now the most common procedures for replanting amputated fingers. When compared to general anesthesia, brachial plexus block anesthesia offers the benefits of a straightforward procedure, a single anesthetic drug, and less interference with the activities of vital organs throughout the body. Furthermore, while maintaining anesthetic safety, the patient may be woken to participate with the surgeon. When compared to local anesthetic, block anesthesia is more comprehensive, has a longer block duration, and the patient can withstand the tourniquet's pain for a longer period of time. Brachial plexus block is still the most used anesthetic approach for finger replantation surgery, despite the use of modern technology such as ultrasonography and nerve stimulators [16]. However, nerve block will still occur in practical practice owing to variables such as the operator's inexperience. The danger of local anesthetic poisoning may be increased simply by raising the dose of local anesthetics. As a result, sedative and analgesic medicines such midazolam, propofol, and sufentanil are often used in clinical settings to increase anesthetic block, although these drugs have side effects include respiratory depression and nausea [17]. Dexmedetomidine provides substantial benefits in conjunction with brachial plexus block during finger replantation due to its unique pharmacological properties.

Dexmedetomidine may be added to postoperative intravenous analgesia pumps for postoperative analgesia in patients with severed digit replantation, in addition to intraoperative use. Continuous dexmedetomidine administration following surgery may help patients achieve sufficient sedative and antianxiety effects, minimise the quantity of opioid analgesics used, limit adverse responses, and improve analgesic effects. Dexmedetomidine mixed with sufentanil has been utilized in the United States for postoperative analgesia in surgical patients, and researchers have discovered that it has a good analgesic effect, minimises adverse responses, improves sleep quality, and lowers stress reactions [18]. As a result, using dexmedetomidine for postoperative analgesia after replantation of severed fingers may enhance sedation and analgesia, minimise the incidence of postoperative adverse events, and raise the replantation of severed fingers survival rate.

## 3. Materials and Method

We selected multiple samples for replantation of amputated fingers. The patients had mild injuries, no hemorrhagic shock and other traumas, and no heart, lung, and other important organ diseases. The American Association of Anesthesiologist (ASA) grade is I-II. All patients were awake, cooperative, coagulation function was normal, neck and shoulder were not damaged or infected, and the anatomical structure was clear. Moreover, all patients did not use analgesia or sedative drugs before the operation, selected brachial plexus block for anesthesia, and signed an informed consent form for anesthesia before the operation. The patients were randomly assigned to one of two groups: ropivacaine mesylate (control group) or dexmedetomidine (treatment group) (test group). The same group of surgeons conducted all of the finger replantation procedures. The average operation time did not vary between the two groups [19].

Criteria for exclusion are (1) the patient is unable to read, comprehend, or communicate; (2) the patient has an ASA of III or higher; (3) the patient has a bleeding tendency or coagulation dysfunction; (4) the patient has a history of local anesthetic allergy, skin infection at the puncture site, or contraindications to regional block anesthesia. Delectation criteria are (1) patients who are not suitable or unable to implement the study plan as planned because of sudden severe complications during the perioperative period (cannot tolerate surgery and anesthesia); (2) patients who need blood product transfusion or continuous pumping of vasoactive drugs to maintain vital signs during surgery; (3) patients need to be transferred to ICU for observation and treatment after surgery; (4) at any stage after entering the study, due to the patient's personal reasons, patients who voluntarily request to withdraw or transfer treatment [20].

Anesthesia: after the patient enters the room, we turn on the anesthesia machine, monitor for self-inspection, and prepare rescue and anesthetic drugs. We need to monitor noninvasive blood pressure (NIBP), heart rate (HR), blood oxygen saturation (SPO2), and electrocardiogram (ECG). At the same time, it is necessary to open a peripheral vein, inject sodium lactate Ringer's solution intravenously, and give midazolam 2 mg intravenously to relieve the patient's nervousness. For brachial plexus block approach, we choose the intermuscular groove. The patient is in a supine position, with his arms flat and close-fitting, his head tilted to the opposite side, revealing the sternocleidomapillary muscles. Later, we found the anterior and middle scalene muscles on the posterior and lateral sides. The space between the two muscles was used as the puncture point at the intersection of the external jugular vein. Then, we used a no. 7 scalp needle to avoid the vertical skin of the external jugular vein and insert the needle slightly to the side of the foot. When the fingers became susceptible, the test group was injected with 20 ml 0.447%ropivacaine mesylate + 0.5 ug.kg − 1 dexmedetomidine mixture, and the control group was injected with 20 ml 0.447% ropivacaine mesylate. During the injection process, it is necessary to observe whether the patient has any abnormal reactions. If the ring and little finger are replanted, axillary sheath nerve block needs to be performed accordingly. The two groups of patients received routine oxygen inhalation by mask during the operation. After the operation, the intravenous self-control pump was turned on, and the two groups had the same formula [21].

The noninvasive blood pressure, heart rate, pulse, and blood oxygen saturation of the two groups of patients were monitored after the block was completed. When the injection is finished, we perform VPS scoring. 0 is painless, mild is 1-3 points, moderate is 4-7 points, and severe is ≥7 points. We took the onset time of blockade from the completion of the injection to pain ≤3 minutes and the time of the anesthesia maintenance time from the completion of the injection to pain sensation >3 and recorded the block onset time and the anesthesia maintenance time of the two groups of patients. At the same time, it is necessary to observe the additional amount of intraoperative local anesthetics, the use of auxiliary analgesics, the analgesic effect of 24 hours postoperatively, and the amount of intravenous self-control drugs used.

## 4. Result

The statistical data in this paper are mainly onset time, anesthesia maintenance time, 24 h analgesic dose, and VAS score (points). The results are shown in Tables 1–4 below, and the corresponding statistical graphs are shown in Figures 1–4.

With the continuous improvement of anesthesia, the two groups of noninvasive blood pressure, pulse, heart rate, and blood oxygen saturation monitoring showed a downward trend, but they were all in the normal range. There were no adverse reactions such as hypotension, bradycardia, and respiratory depression. In comparison between groups, the test group is lower than the control group, *P* > 0.05, which is not statistically significant. When the onset times of the two groups are compared, the test group is quicker than the control group, with a statistically significant difference of *P*0.05. When comparing the duration of action across groups, the test group outlasts the control group by a statistically significant margin. In comparison to the other two groups, the blocking effect is pretty perfect. Furthermore, no further analgesics or local anesthetics are used. The surgeries were finished in 6 hours, and all of the patients fell asleep peacefully after being given 2 mg of midazolam. Intraoperative analgesia is adequate, muscle relaxation is adequate, blood vessels are dilated, and tendon tension is minimised, resulting in favourable surgical settings. When comparing analgesic effects 24 hours after surgery, the test group's dosage of analgesic medicines is lower than the control group's, and the difference is statistically significant. The test group outperforms the control group in terms of VAS scores, and the difference is statistically significant. On the basis of the above experiments, the patient's rehabilitation effect and patient satisfaction are counted, and the results obtained are shown in Table 5, Table 6, Figures 5 and 6.

It can be seen from the above studies that the recovery effect and patient satisfaction of the test group are higher than those of the control group.

## 5. Conclusion

The replantation of severed finger takes a long time, the operation is delicate, and the requirement for anesthesia is high. It is difficult to meet the requirements of nerve block using local anesthetics alone. In addition to intravenous infusion, dexmedetomidine can also be used as a local anesthetic adjuvant to enhance anesthesia. Alpha2-adrenergic receptor agonists have sedative, antianxiety, hypnotic, analgesic, and sympathetic effects. Dexmedetomidine is a highly selective *α*2-adrenergic receptor agonist, which is 1600 times more selective for *α*2 receptors than *α*1 receptors.

Dexmedetomidine has been utilized as an auxiliary medication for central and peripheral nerve block in recent trials and has shown to be effective. In this research, the control group had a much shorter start time and a significantly longer action period than the observation group. The efficacy of dexmedetomidine as an adjuvant for ropivacaine mesylate is clear. In the replantation of severed fingers, preventing vasospasm is a tough task. A good and long-lasting brachial plexus block may successfully avoid vasospasm caused by pain by blocking sympathetic nerves for a long time, keeping blood vessels dilate. It may also improve blood flow, enable tissue perfusion and vascular anastomosis, avoid arteriovenous thrombosis caused by vascular anastomotic stenosis, delay blood flow, and platelet aggregation, and lessen limb restlessness-related problems. Hypotension, hypertension, bradycardia, and respiratory depression are among side effects of dexmedetomidine. The most common cause is a single intravenous injection or an overdose. There was no evident cardiovascular reaction or respiratory depression in this research. Dexmedetomidine may be in a small dose, mainly distributed around the nerves, and the blood concentration is low. Therefore, there are fewer adverse reactions.

## Figures and Tables

**Figure 1:** Statistical results of onset time.

**Figure 2:** Statistical results of anesthesia maintenance time.

**Figure 3:** Statistics results of 24 h analgesic drug dosage.

**Figure 4:** Statistical results of VAS score.

**Figure 5:** Statistical results of rehabilitation effects.

**Figure 6:** Statistical results of patient satisfaction.

**Table 1:** Statistical table of onset time.

Number	Control group	Test group	Number	Control group	Test group	Number	Control group	Test group
1	10.96	8.35	13	11.55	6.00	25	16.73	5.03
2	10.67	6.74	14	16.19	9.27	26	10.90	10.61
3	17.84	6.79	15	11.75	6.62	27	15.42	9.54
4	17.86	9.27	16	10.92	9.40	28	14.81	4.71
5	17.03	6.62	17	16.58	10.26	29	16.30	10.14
6	17.53	10.02	18	13.89	9.41	30	15.62	10.19
7	14.47	4.93	19	12.89	5.13	31	14.16	7.17
8	12.25	9.31	20	16.20	10.26	32	12.54	4.93
9	10.36	9.38	21	14.50	5.57	33	17.79	7.99
10	11.00	10.40	22	15.89	9.04	34	14.92	8.21
11	11.83	5.19	23	18.40	7.67	35	17.48	7.27
12	11.45	5.86	24	15.66	8.10	36	16.16	8.24

**Table 2:** Statistical table of anesthesia maintenance time.

Number	Control group	Test group	Number	Control group	Test group	Number	Control group	Test group
1	451.51	673.67	13	378.85	708.01	25	432.53	611.57
2	423.51	610.00	14	462.91	695.11	26	413.80	745.90
3	341.05	711.14	15	323.75	657.25	27	452.56	808.92
4	477.27	531.20	16	389.40	564.45	28	420.47	545.19
5	457.56	764.06	17	478.65	588.83	29	489.03	599.71
6	555.09	626.14	18	363.72	743.36	30	371.07	752.84
7	432.54	581.17	19	326.76	549.47	31	509.68	733.65
8	552.33	692.11	20	510.07	749.41	32	478.29	541.17
9	331.51	539.28	21	534.35	557.86	33	560.56	722.46
10	328.66	616.96	22	473.26	601.56	34	461.12	674.66
11	460.97	824.12	23	409.61	621.72	35	456.79	813.87
12	496.80	613.73	24	544.57	601.49	36	335.75	607.51

**Table 3:** Statistical table of 24 h analgesic drug dosage.

Number	Control group	Test group	Number	Control group	Test group	Number	Control group	Test group
1	54.43	38.02	13	53.84	38.77	25	52.39	38.72
2	53.80	41.44	14	56.42	38.40	26	54.21	43.91
3	57.45	43.99	15	51.99	41.70	27	51.00	41.26
4	55.81	38.71	16	54.02	42.54	28	53.35	39.31
5	53.92	41.76	17	53.73	41.72	29	51.44	42.03
6	49.93	38.48	18	55.38	43.33	30	52.95	42.60
7	52.92	41.72	19	55.04	41.01	31	57.12	39.95
8	52.30	41.32	20	48.59	39.30	32	49.46	38.74
9	55.47	43.10	21	53.24	39.82	33	54.52	43.87
10	55.49	43.33	22	56.61	42.01	34	49.97	39.45
11	52.48	39.43	23	51.51	43.93	35	50.50	38.48
12	57.34	42.64	24	49.90	42.34	36	57.72	41.23

**Table 4:** Statistical table of VAS score.

Number	Control group	Test group	Number	Control group	Test group	Number	Control group	Test group
1	2.00	0.70	13	2.35	0.53	25	1.88	0.72
2	2.09	0.64	14	2.50	0.87	26	2.05	0.97
3	1.66	0.53	15	1.35	0.57	27	2.37	0.40
4	2.05	0.53	16	1.88	0.90	28	1.71	0.80
5	2.11	0.75	17	1.56	0.77	29	2.46	0.96
6	1.87	0.68	18	1.62	0.59	30	2.75	0.88
7	1.40	0.54	19	2.14	0.49	31	1.68	0.43
8	2.52	0.67	20	1.52	0.99	32	1.72	0.41
9	1.57	0.53	21	1.92	0.67	33	1.47	0.94
10	2.68	0.81	22	2.17	0.65	34	1.24	0.74
11	2.32	0.79	23	2.31	0.46	35	2.10	0.71
12	1.68	0.52	24	1.44	0.68	36	1.65	0.81

**Table 5:** Statistical table of rehabilitation effect.

Number	Control group	Test group	Number	Control group	Test group	Number	Control group	Test group
1	91.24	96.29	13	84.57	90.87	25	87.34	95.77
2	91.30	96.72	14	85.43	93.59	26	84.04	88.01
3	91.22	88.29	15	89.62	88.96	27	89.07	95.56
4	90.74	93.25	16	91.81	96.96	28	92.19	90.42
5	91.85	92.12	17	91.72	89.59	29	87.59	96.36
6	87.37	88.59	18	84.14	90.18	30	84.73	90.10
7	84.43	91.64	19	88.01	91.71	31	86.63	92.79
8	85.97	88.45	20	92.55	95.81	32	87.72	97.57
9	85.57	90.26	21	88.52	94.38	33	93.41	97.01
10	85.49	95.30	22	84.58	88.67	34	84.29	90.77
11	86.81	97.81	23	88.12	93.41	35	93.79	93.10
12	84.03	95.96	24	85.85	89.74	36	85.48	97.89

**Table 6:** Statistical table of patient satisfaction.

Number	Control group	Test group	Number	Control group	Test group	Number	Control group	Test group
1	85.95	95.06	13	90.95	96.27	25	91.87	89.11
2	88.06	93.70	14	93.87	96.14	26	86.01	89.53
3	86.57	89.85	15	89.51	92.76	27	89.32	88.94
4	86.99	97.63	16	87.42	90.66	28	92.61	88.30
5	86.72	89.92	17	87.36	93.17	29	84.19	92.08
6	90.71	93.99	18	93.40	90.58	30	91.73	92.65
7	90.20	92.14	19	86.66	88.22	31	87.57	88.62
8	88.16	96.89	20	84.30	97.35	32	84.99	94.20
9	86.89	92.91	21	88.84	89.79	33	84.21	92.08
10	90.33	97.38	22	93.92	88.18	34	86.34	94.41
11	87.72	92.41	23	93.95	89.20	35	84.62	89.36
12	88.11	93.19	24	87.53	97.61	36	84.92	95.12

## Data Availability

The data used to support the findings of this study are included within the article.
